The article "Anthropological responses to environmental challenges in SAARC nations: A comparative analysis" was retracted in 2025. Reasons: concerns about the peer review; concerns about the authorship.

# Anthropological responses to environmental challenges in SAARC nations: A comparative analysis

**DOI:** 10.1371/journal.pone.0296516

**Published:** 2024-02-08

**Authors:** Chunyan Liu, Muneeb Ahmad, Ali Altalbe

**Affiliations:** 1 School of Community for Chinese Nation, North Minzu University, Yinchuan, Ningxia, China; 2 Jiangxi University of Finance and Economics, Nanchang Jiangxi, China; 3 Department of Computer Engineering, Prince Sattam bin Abdulaziz University, Al-Kharj, Saudi Arabia; 4 Faculty of Computing and Information Technology, King Abdulaziz University, Jeddah, Saudi Arabia; Second Xiangya Hospital, Central South University, CHINA

## Abstract

The purpose of the study is to investigate the relationships and potential impacts of environmental pollutants, human resources, GDP, sustainable power sources, financial assets, and SAARC countries from 1995 to 2022. Board cointegration tests, D-H causality, cross-sectional reliance (CSD), Saville and Holdsworth Restricted (SHL), and the DSK Appraisal Strategy were among the logical techniques employed to discover long-term connections between these components. Results demonstrate that GDP growth, renewable energy sources (REC), and environmental pollution (ENP) all contribute to SAARC countries’ progress. However, future opportunities and HR are negatively impacted by increased ecological pollution. The results of the two-way causality test demonstrate a strong correlation between HR and future possibilities. Opportunities for the SAARC countries are closely related to the growth of total national output, the use of green electricity, and public support sources. Ideas for tackling future projects are presented in the paper’s conclusion. These include facilitating financial development, reducing ecological pollution, financing the progress of human resources, and promoting the use of sustainable power sources.

## 1. Introduction

According to the latest assessment study from the International Panel on Climate Change (IPCC), human-caused natural changes are already having an impact on a wide range of climate and ecological variables on a global scale [1]. Worldwide, air pollution is responsible for a significant number of avoidable deaths annually, according to World Health Organization (WHO) estimates [2]. Whether environmental contamination poses a serious threat, perspectives like health, availability of clean water, and improved sanitation shape future possibilities. There is a unidirectional causative relationship between the negative impacts of petroleum derivatives and future problems with environmental pollution, but a bidirectional causal relationship between disinfection and water use [3]. According to [4], a good percentage of a population’s health is predicted by its future, or the average number of years people expect to live. According to [5], there is a strong correlation between financial development and longer futures. Real wages and the use of renewable energy sources have a significant impact on the future. Better access to healthcare, made possible by rising wages from a more developed human resource sector, increases future earnings [6]. In comparison to petroleum products, renewable energy sources contribute less to air pollution and increase the time that humans may expect to live on earth [7]. The positive effects of salary levels more than compensate for the negative effects of public sustainable power in the future. Reducing resource usage and environmental pollution are two goals of environmental laws [8]. It is possible to compare the SAARC countries’ futures with those of other groups, such as those concerned with human capital, ecological manageability, sustainable electricity use, natural pollution, and GDP growth. The experts used logical procedures such as the Saville and Holdsworth Confined (SHL) tests, cross-sectional reliance (CSD), and the Driscoll and Kraay (DSK) mistake approach to analyze the collected data. With a proportionate relationship between HC and LE, which features the meaning of equal access to medical care and education, solid clinic medical care frameworks are vulnerable to GDP development and monetary turn of events. To increase both financial and human resources, it is essential to create an environment that is optimal for health improvement. Environmental pollution and the use of green electricity led to cleaner circumstances, which have a significant impact on both the immediate and distant future. Both good and bad natural quality shocks cause future reactions to change. The assessment settles on the conclusion that switching to greener power sources ensures better energy efficiency and financial performance, helps reduce CO_2_ emissions, and has no negative impact on GDP growth. The use of renewable energy sources is inversely proportional to long-term trends in environmental pollution and positively correlated with GDP growth and decline.

The article "Anthropological responses to environmental challenges in SAARC nations: A comparative analysis" was retracted in 2025. Reasons: concerns about the peer review; concerns about the authorship.

The second part of the evaluation is a study of written work that concludes earlier research to highlight the relevance of the current investigation. In Section 3, the econometric model approach is shown from top to bottom. In Section 4, backed by tables and statistics, are the results and defenses. Sections 5 provides a detailed discussion of the results.

## 2. Literature review

The complex relationship between financial progress and an enlarged future, showing a positive correlation between the two, is due to several factors [9]. This relationship is bolstered by improved access to healthcare, sanitary living circumstances, good direction, and educational opportunities within networks [10]. Increases in GDP make the construction of robust healthcare infrastructure, such as hospitals and clinics, more feasible [11]. A better future is possible because education equips individuals with knowledge of healthy living, disease prevention, and expanded business opportunities [12]. Both the immediate and distant futures are profoundly impacted by the use of renewable energy sources in proximity to petroleum derivatives [13]. In general, it could be worth it to trade an additional year in the future for about 9% of annual customer expenditure. Even if economic growth increases life expectancy, the negative health effects of delayed exposure to pollution and environmental hazards may cancel each other out [14]. Education has a key role in the future since it leads to better lifestyles and more autonomy, which in turn expands opportunities [15]. Healthcare, prevention, and wellness innovation initiatives are thought to be the driving forces behind future growth [16]. Proficient clinical interventions and illness prevention, as part of a robust healthcare system, lead to improved long-term health outcomes [17]. Human Resources, via education and job experience, opens doors to financial opportunities [18]. Improving human resources and prospects requires resolving health disparities, creating an environment conducive to lifelong learning, and ensuring equal access to medical treatment and education [18]. Highlighting the link between environmental pollution and its consequences, the article highlights the negative impact of ongoing contamination on future events [19]. Hazardous compounds in water bodies are identified as threats to human health. Synthetics that deplete the ozone layer contribute to climate change, which has negative effects on human health and other biological systems [20]. The introduction of gases and other human activities amplifies the nursery effect and contributes to the hazardous atmospheric deviation [21]. Renewable energy sources, such as solar, wind, hydropower, and geothermal heat, produce fewer ozone-depleting pollutants than traditional power plants [22]. By reducing air pollution, adopting renewable energy sources helps create cleaner environments, which has far-reaching consequences for the future [23]. Improvements in practical electricity, especially in areas not connected to the network, provide basic services like medicine and vaccine refrigeration and illumination [24]. Supportable power company development leads to job openings, monetary development, and less reliance on non-sustainable power sources imported from outside [25]. The well-being and integrity of a community are impacted by the mining and management of common resources. Improving transportation organizations and framework projects is a common outcome of resource extraction, which often leads to financial recirculation and enlarged company potential opportunities [26]. According to [27] managing resource exploitation is crucial for maximizing benefits while minimizing drawbacks. However, the covert health applications disrupt economic growth and cause a 1% increase in mortality rates in the future [28].

The article "Anthropological responses to environmental challenges in SAARC nations: A comparative analysis" was retracted in 2025. Reasons: concerns about the peer review; concerns about the authorship.

## 3. Research methodology

### 3.1 Data collection

Table 1 considers the variable’s issues in the context of data from 1995 to 2022, which includes Afghanistan, Bangladesh, and the SAARC countries (Nepal, India, Bhutan, Sri Lanka, and Pakistan). The SAARC countries have been treated unfairly when selecting the study, given how natural it is to achieve proof. Future calculations are strong as they enter the world every year that is possible, and they are seen as a consistent measure of overall well-being.

**Table 1:** Description of variables.

Symbols	Variable	Details	References
LE	Life Expectancy	Future healthcare services and people’s aspirations for basic conveniences	https://data.worldbank.org.com
GDP	GDP Growth	Overall production in the country	https://data.worldbank.org.com
REC	Renewable Energy Consumption	Renewable energy sources include biomass, geothermal heat, solar power, and wind power.	https://www.imf.org.com
HC	Human Capital	The power of people, or human resources	https://data.worldbank.org.com
ENP	Environmental pollution	One major source of environmental pollution is carbon dioxide.	https://data.worldbank.org.com
ENS	Economic and Natural Sources	ENS controls Standard Monetary Sources of Rent as a percentage of GDP	https://www.imf.org.com

### 3.2 Econometric model

The study has followed [29], who developed models of medical care and well-being to identify certain attributes as key components of a compelling future (LE) among the SAARC countries. The material was thoroughly verified using the DSK Assessment Strategy, the Saville and Holdsworth Restricted (SHL) test, Dumitrescu and Hurlin’s CSD and D-H causality tests. The study elements in Eq 1 is presented to determine the role of the LE antecedent.


$$\text{LE}=\left(\text{REC},\text{ENP},\text{GDP},\text{ENS},\text{HC}\right)$$ (1)

Eq 2 expresses the logarithm limit between the segments subsequently about time has approved.


$${\text{lnLE}}_{it}=\Omega_{i}+{\text{glnREC}}_{it}+{\text{hlnENP}}_{it}+{\text{ilnGDP}}_{it}+{\text{jlnENS}}_{it}+{\text{klnHC}}_{it}+\epsilon_{it}$$ (2)

Where the “ln” is the logarithm function, “Ω” is the constant function, “g” to “h” show the coefficients of regressions, and “ϵ” denotes the error term.

The article "Anthropological responses to environmental challenges in SAARC nations: A comparative analysis" was retracted in 2025. Reasons: concerns about the peer review; concerns about the authorship.

#### 3.2.1 SHL and CSD tests

Board information concerns, such as their potential geological spread, unexplained portions, and continuous connections, maybe more easily identified and resolved with the use of the Saville and Holdsworth Restricted (SHL) and Cross-Sectional Reliance (CSD) testing. As seen in Eq 3, the CSD keeps universal econometrical competencies.


$${\left(CSD\right)}_{rs}=\Sigma_{j=1}^{m-1}\Sigma_{i=j+1}^{m}{\overset{ˇ}{\rho }}_{ij}^{2}$$ (3)

The CSD test-scaled LM, shown in Eq 4, is the all-inclusive test measurement that makes use of distinct model bounds [32].


$${\left(CSD\right)}_{lm}=\sqrt{\frac{1}{m(m-1)}}\;\sum_{j=1}^{m-1}\sum_{i=j+1}^{m}{\overset{ˇ}{\rho }}_{ij}^{2}$$ (4)

If the time interval in Eq 5 is not indeed the cross-sectional area, an additional CSD test that is used statistically is Pesaran’s (2007) CSD test.


$$(CSD)=\sqrt{\frac{1}{m(m-1)}}\Sigma_{j=1}^{m-1}\Sigma_{i=j+1}^{m}{\overset{˘}{\rho }}_{ij}^{2}$$ (5)

The CSD test developed by [30] is also applied in Eq 6.


$$CSD_{LM}=\sqrt{\frac{1}{m(m-1)}}\sum_{j=1}^{m-1}\sum_{i=j+1}^{m}\;{\overset{ˇ}{\rho }}_{ij}^{2}-1-\frac{m}{2(s-1)}$$ (6)

The deviation from the OLS for SAARC countries is denoted by ${\overset{ˇ}{\rho }}_{ij}^{2}$. Although the ’s’ presents the cross-sectional area, the ’m’ suggests a period. Eq 7 and 8 provides the configuration of SHT, according to the evaluation of [31].


Δ^SHT=m1/2.2y−1/2řm1−y) (7)

Δ^A∘SHT=m1/2⋅2y−1/22m(r−y−1r+1−1/2řm1−y) (8)

The delta of the $\hat{\Delta }$SHT is represented by ΔSHT, while the identifiable SHT is denoted by $\hat{\Delta }\overset{\circ }{\text{A}}$SHT.

#### 3.2.2 CIPS and CADF outcomes

The two most recent second-generational stationarity approaches are used to analyze the limits, and the CADF and CIPS trials of [32] have been used for stationarity. When compared to more conventional methods, these stationarity-based approaches perform better when assessing and correcting CSD exceptions in the board dataset [33]. The initial unit root test was not as solid or accurate as these fixed procedures [34]. The mathematical solutions to the two tests are in Eqs 9 and 10.


$$(CADF)=\varpi y_{it}=\beta_{it}+x_{it-1}+\Omega_{I}\text{s}+\sum_{i=1}^{m}\varpi_{ij}\varpi y_{jt-i}+\epsilon_{it}$$ (9)

Such that “ω” signifies the alterations between the variable, “x*_it_*” the examination sequences.


$$\text{CIPS}=\frac{1}{n}\;\sum_{i=1}^{n}\Omega_{i}(n,S)$$ (10)

The above equation shows that “s” signifies the cross-sections and “m” stands period dated.

The article "Anthropological responses to environmental challenges in SAARC nations: A comparative analysis" was retracted in 2025. Reasons: concerns about the peer review; concerns about the authorship.

#### 3.2.3 Cointegration test

The SHT and CSD tests in the exploration model were controlled using the [35] cointegration test. The board examination test (*H*_τ_—*H*_*a*_) and the crowd valuation test $\left(H_{k}-H_{\alpha }\right)$ a are the two types are covered in Eqs 11 to 14.


$$H_{\kappa }=\frac{1}{n}\;\sum_{i=1}^{m}\frac{\delta_{i}}{s.e\left({\hat{\delta }}_{i}\right)}$$ (11)

$$H_{\alpha }=\frac{1}{m}\;\sum_{i=1}^{m}\frac{s\delta_{i}}{1-\sum_{j=1}^{k}\;{\hat{\delta }}_{ij}}$$ (12)

$$R_{\kappa }=\frac{\delta_{i}}{s.e\left({\hat{\delta }}_{i}\right)}$$ (13)

$$R_{\alpha }=\text{s}\delta_{i}$$ (14)

The “*δ*_*i*_” expressions the variations reliability.

#### 3.2.4 DSK’s rate outcomes

According to [36], the evaluation makes use of the DSK valuation technique, which is a quantifiable way to measure the standard errors in relapse models for board data and uses a weighting scheme to alter the covariance framework first presented in Eq 15.


$$Y_{it}={\text{Y}}_{it-1},c+{\text{x}}_{it}\text{y}+\varepsilon_{it}\;i=1,\ldots ,\text{m},\text{T}=1,\ldots \text{s}$$ (15)

The *Y*_*it*_ expresses the life expectancy, X_*it*_ displays the regressors (*REC*, *HC*, *ENS*, *GDP*, *and ENS*).

#### 3.2.5 Robustness analysis

Two sorts of econometrics are utilized to test the power of the DKS technique. The AMG and CCE-MG strategies are intended to represent these unnoticed heterogeneities and give more hearty assessments in board settings. Board information AMG and CCE-MG approaches handle sequential relationships, autocorrelation, and unnoticed heterogeneity [37].

### 3.3 Scrutiny of causality test

The study uses the D-H causality test, to determine the strength of the components’ clear associations with one another. It is a novel approach, however, previous research has used the DH system to examine the relationships between different data sets [38], as defined in Eq 16.


$$Y_{it}=\alpha_{i}+\sum_{m=1}^{M}\Omega_{j}^{m},Y_{j(m-t)}+\sum_{m=1}^{M}\varphi_{j}^{n},X_{j(n-t)}$$ (16)

## 4. Results and discussions

### 4.1 Descriptive statistics

The explicit measurements, connection tests, and VIF analyses of the study factors are shown in Table 2.

**Table 2:** Descriptive, bivariate correlation, and multicollinearity analysis.

Variables	LE	GDP	ENP	HC	REC	ENS
Mean	57.187	22.281	11.987	0.479	1.975	1.992
Median	64.382	23.528	12.876	0.623	2.821	1.923
SD	2.989	0.632	0.855	0.315	0.398	1.697
Max.	78.996	29.689	13.986	1.968	3.955	3.852
Min.	48.852	21.875	10.679	0.462	2.568	2.973
Skewness	-0.387	-0.429	-0.423	-0.648	0.247	-0.632
Kurtosis	3.989	2.004	1.956	3.024	2.000	2.028
Jarque-Bera estimate	0.0122	5.856	9.2565	14.985	2.998	10.235
Probability	0.0021	0.0001	0.0000	0.0001	0.0002	0.0000
***Bivariate correlation analysis using Pearson’s tau***						
LE	1					
GDP	0.601***	1				
ENP	0.472	-0.498***	1			
HC	0.510	0.298	0.398***	1		
REC	0.376	0.402	0.537	0.529***	1	
ENS	-0.418	-0.398	-0.259	-0.523	0.601	1
***variance inflation factor analysis***						
***Variable***	***VIF***		***Tolerance = 1/VIF***			
LE	1.956		0.532			
GDP	1.909		0.403			
ENP	1.978		0.398			
HC	4.001		0.321			
REC	2.988		0.389			
ENS	3.526		0.302			

Note: ***p<0.001. REC: renewal energy consumption, LE: life expectancy, GDP: gross domestic production, ENC: economic natural resources, HC: human capital, VIF: variance inflation factor,

Connectivity tests are used to find connections between components to ensure that coefficient gauges are accurate. VIF focuses on examining multicollinearity in relapse models. The study’s findings revealed clear causal links between the variables. Specifically, the study found that ENP, ENS, and LE had an inverse association with one another. When normal financial assets become less accessible, future increases occur [39]. Multicollinearity, as seen in Fig 1, affects the reliability of the relapse study because of the strong relationships between the indicator variables.

The article "Anthropological responses to environmental challenges in SAARC nations: A comparative analysis" was retracted in 2025. Reasons: concerns about the peer review; concerns about the authorship.

**Fig 1:** Presents the trend assessments of economic natural resources in the SAARC countries.

VIFs are below the specified removal value since multicollinearity is reduced with lower VIF values [40]. Although the VIF test is useful for identifying multicollinearity, it isn’t the only factor that determines whether a relapse model is valid. The results show that, similar to [41] found, REC, HC, and GDP were seen as strongly linked to the future.

### 4.2 Investigative CSD and SHT

The board dataset’s erroneous hypothesis is categorically rejected by the financial elements evaluated by CSD assessment procedures. Using CSD evaluation procedures to survey financial elements leads to an examination that is headed by SHT tests at the base, which deny slant homogeneity; the fallacious supposition is mixed by the (SHT) test. To measure the impact of the study’s variables, researchers use a trustworthy method known as the CSD assessment technique. Table 3 represents the several financial factors will shape in the future.

**Table 3:** Represents the results of the SHT and CSD test.

*Variables*	*Bias-Corrected Scaled LM*	*Pesaran’s LM*	*Breusch-Pagan LM*	*Pesaran’s CD*
ln (LE)	35.011***	35.897***	129.871***	11.029***
ln (GDP)	46.238***	51.024***	159.998***	12.054***
ln (ENP)	35.021***	32.058***	118.904***	6.056***
ln (HC)	42.598***	42.002***	165.035***	11.085***
ln (REC)	23.002***	21.026***	129.024***	10.985***
ln (ENS)	32.987***	32.068***	142.053***	9.897***
***Slope Homogeneity Test results***				
*Delta tilde* Δ	11.033***			
*Delta tilde adjusted*Δ	12.989***			

There was no issue of CSD as a result of a board dataset that used a cross-sectional dependence assessment technique, which was a deceptive assumption. Findings highlight the significance of taking interdependencies and heterogeneity into account when examining the relationships within the board dataset [42]. One way to measure the consistency with which factor-to-factor correlations follow expectations over time is with the SHT (Slope Homogeneity Test).

The article "Anthropological responses to environmental challenges in SAARC nations: A comparative analysis" was retracted in 2025. Reasons: concerns about the peer review; concerns about the authorship.

### 4.3 CIPS and CADF evaluations

The stationarity get together between the study factors is laid out in Table 4, which covers the CADF and CIPS approaches. The variables in a board dataset can be either fixed or coordinated using cross-sectional Im-Pesaran-Shin (CIPS) board unit root tests or cross-sectional extended Dickey-Fuller (CADF) tests.

**Table 4:** The results of CADF and CIPS tests.

Variables		CADF		CIPS	
	*Exercise of Integration*	*Level*	*1*^*st*^ *Difference*	*Level*	*1*^*st*^ *Difference*
ln(LE)	I (1)	-0.39	-5.204***	-1.184	-4.274***
ln(GDP)	I (1)	-2.014	-5.099***	0.581	-4.351***
ln(ENP)	I (1)	-1.434	-4.943***	1.994	-4.512***
ln(HC)	I (1)	1.043	-5.148***	-0.344	-5.135***
ln(REC)	I (1)	1.897	-9.235***	-0.914	-9.217***
ln(ENS)	I (1)	-0.589	-9.931***	-0.444	-5.468***

A consistent correlation between the study criteria is revealed by the results. The first request, or I(1), coordinates the period series model’s borders. The ln(LE), ln(GDP), ln(ENP), ln(HC), ln(REC), and ln(ENS) all have present-day stationarity relationships. The unit root invalid conjecture is tested for stationarity using the CADF test. Im-Pesaran-Shin is utilized in CIPS, another board unit root test, to assess cross-sectional dependency [43].

### 4.4 Inspection for board cointegration

Presented in Table 5 are the outcomes of the board cointegration test. Before dissecting the long-term impacts of ln(LE) and ln(GDP), ln(ENP), ln(HC), ln(REC), and ln(ENS) on ln(LA), it is crucial to verify that cointegration is feasible in the exploration model. Both the bunch insights classification (*G*_*t*_−*G*_*a*_) and the board examination classification (P_*t*_ − *P*_*a*_) confirmed that the series under scrutiny had long-term relationships.

**Table 5:** The cointegration test outcomes.

	*Value*	*Standardized estimate*	*Significance*
Q*c*	-4.498	2.246	0.839
Q*α*	-6.442***	4.471	0.001
H*c*	-5.049	2.398	0.046
H*α*	-6.982***	4.008	0

Note: *** p < 0.001

The study rejects the false hypothesis at the 1% level of significance. According to [44], there was a strong correlation between the population and the future life expectancy in short-run. A 1% significance level indicates a high degree of confidence in ignoring the unfounded conjecture.

The article "Anthropological responses to environmental challenges in SAARC nations: A comparative analysis" was retracted in 2025. Reasons: concerns about the peer review; concerns about the authorship.

### 4.5 Approximations of the DSK test

Results from the DSK inquiry test on the effects of HC, REC, ENP, and ENS on LE, as well as gross domestic product development, have been analyzed. Table 6 represents the findings of the DSK inquiry tests for SAARC countries.

**Table 6:** The DSK analysis test outcomes.

*Variables*	*Estimate*	*SE*	*Significance*
ln (LE)	0.251***	0.021	0.0001
ln (GDP)	-0.298***	0.026	0.0000
ln (ENP)	0.325***	0.652	0.0000
ln (HC)	0.532***	0.047	0.0000
ln (REC)	-0.219***	0.037	0.0006
Persistent	4.212***	0.712	0.0002
***Investigation***			
R^2^	0.705	Jarque Bera test	7.019 (0.427)
Adj-R^2^	0.691	Wald test	201.022 (0.020)
F-value	215.175***	Wooldridge test	522.070 (0.772)
Significance	0.0000		

Note: *** p<0.001.

A 1% increase in GDP further improves LE in SAARC countries, since the gross domestic product coefficient metric is large and positive at the 1% significance level. The growth of SAARC nations’ gross domestic output helps them to further expand their health use. Residents become more health conscious, alter their comfort assumptions, and ultimately improve LE as a result of higher wages and GDP. According to the results, the GDP development has a strong and negative effect on LE, and according to DSK testing, CO_2_-assessed ENP is inversely related to LE. Increasing ENP by 1% reduces LE, and CO_2_ emissions pollute the air, which harms human health and reduces LE, according to [45]. Medical care, security, and financial obligations are provided by the administrators of these nations with larger gross domestic product [46]. Gross domestic product growth leads to higher rent, which stabilizes people’s finances and makes it possible for them to pay for quality clinical healthcare [47]. The results demonstrate that the most definite variable impacting human health is frequent pollution, and the LE of SAARC residents are affected by HC increases brought about, and it is confirmed by [48]. According to [49], human resource interests have a significant impact on wellbeing outcomes. However, financial potential and human resource enhancement are hindered by chronic fragility. According to [50], people’s health issues are impacted by their level of training in a multiplicative manner. In SAARC nations, the DSK model studies have shown that REC is beneficial and primarily impacts LE, with a 1% increase in REC positively impacting LE [51]. A non-REC-producing approach produces toxins that endanger human life, whereas the REC further develops LE decisively [52]. The DSK method found that in the SAARC region, ENS and LE are inversely associated, for every one percent increase in ENS extraction, there is a one percent decrease in LE [53].

The article "Anthropological responses to environmental challenges in SAARC nations: A comparative analysis" was retracted in 2025. Reasons: concerns about the peer review; concerns about the authorship.

### 4.6 Robustness analysis

Researchers and politicians in the SAARC countries depend on the strength assessment to provide the right guidelines for growing LE, and the assessment is quantitatively sound. Table 7 represents the DSK method that agrees with the AMG and CCEMG coefficient evaluations. The findings corroborate the audit’s conclusions of SAARC countries’ LE’s primary factors.

**Table 7:** The robustness analysis test outcomes.

*Variables*	*CCEMG*		*AMG*	
	*Coefficient*	*Significance*	*Coefficient*	*Significance*
ln (GDP)	0.479***	0.0002	0.272***	0.0000
ln (ENP)	-0.304***	0.0001	-0.430***	0.0020
ln (HC)	0.207***	0.0022	0.053***	0.0022
ln (REC)	0.021***	0.0004	0.972***	0.0040
ln (ENS)	-0.076***	0.0010	-0.264***	0.0000
*R* ^2^	0.406			
Adjusted *R*^2^	0.716			

Note: *** p < 0.001

The power test of the SAARC countries revealed several significant future-influencing elements. Progress in these areas includes things like population growth, renewable energy, public funding, human capital, and GDP. Higher rates of gross domestic product development are frequently associated with more notable investments in social administrations such as healthcare and education, which can benefit the future. In this context, "human resources" refers to the workers’ knowledge, skills, and well-being. The health care and general development systems of a country benefit from its access to various financial assets. Jakovljevic et al. (2020) [54] found that the future and wellness results are affected by population thickness and levels of urbanization. Reduced air pollution and improved overall health are long-term effects of increased access to renewable energy.

### 4.8 Influential derivation and significance

Despite highlighting the connection, assessment methods such as DSK, AMG, and CCEMG fail to demonstrate a causal relationship between the variables. Therefore, to determine if systemic implications for one macroeconomic indicator impact another, a causality test should be conducted. This study looked at the D-H method proposed by Dumitrescu and Hurlin, for determining the causes of interface events [55]. Table 8 displays the results of the paper’s causality analysis. The study found a one-way relationship between the GDP, REC, ENS, and LE of the country. Since these foci are related under two domains, the ENP and HC technique plans should include an LE-further developing methodology.

**Table 8:** The D-H causality test outcomes.

Null Hypothesis	W-value	Zbar-value	p-value	Observations
LnGDP ⇎ LnLA	5.715***	4.559	0.0000	GDP →LA
LnLA ⇎ LnGDP	2.437	0.449	0.0039	
LnENP ⇎ LnLA	9.565***	9.052	0.0000	ENP ⟷ LA
LnLA ⇎ LnENP	4.729***	4.209	0.0001	
LnHC ⇎ LnLA	4.311***	4.325	0.0024	HC ⟷ REC
LnLA ⇎ LnHC	7.024***	2.198	0.0010	
LnREC⇎ LnLA	4.521***	5.301	0.00046	REC → LA
LnLA ⇎ LnREC	2.098	0.348	0.00356	
LnENS ⇎ LnLA	5.474***	4.442	0.0002	ENS →LA
LnLA ⇎ LnENS	2.424	0.437	0.4490	

Note: *** p < 0.001.

The article "Anthropological responses to environmental challenges in SAARC nations: A comparative analysis" was retracted in 2025. Reasons: concerns about the peer review; concerns about the authorship.

Air and water pollution are examples of environmental contaminants that harm human health. Exposure to toxic substances can cause a variety of health problems, including respiratory and cardiovascular diseases, which can shorten a person’s lifespan. In addition, biological systems and biodiversity are negatively impacted by natural pollution, which in turn impacts human well-being [56]. There is a strong relationship between environmental pollution, human resources, and social orders’ ability to monitor clinical difficulties and adopt improved habits [57]. Researchers should also consider the inverse relationship between biological degradation and human resources.

### 4.9 Discussions

The results of the study reveal several noteworthy relationships between different factors and potential outcomes. HC, ENP, ENS, and REC are linked to what’s to come in the future. The diversification of China’s goods has led to a decline in CO_2_ emissions [58]. Greater GDP, HC, ENS, and REC are all indicators of an expanding future. The assessment concludes that future success is due to increased financial development, better human resources, the use of sustainable assets, and the use of sustainable power sources. Reduced long-term environmental damage from an expanding economy is one benefit of sustainable power [59]. Although GDP increases pollution outflows, slowing economic development, HC and ENP affect LE [60]. Less human resources and more contaminants mean fewer futures. Because economic growth and environmental pollution affect people’s health, the causality focus identified a one-way relationship between past events, present conditions, and future sustainability in power consumption [61]. A more remarkable future is the result of increased financial success and the use of renewable power sources. No evidence has been found to suggest a negative correlation between the long-run and financial growth. [62] found that organizing environmentally friendly power sources is an effective strategic tool for reducing emissions of ozone-harming compounds that do not impede economic growth. Supporting sustainable power sources, reducing pollution, investing in human resources, and advancing economic growth are all ways to increase life duration. According to [63], the development of gross domestic product is positively correlated with fossil fuel byproducts. Despite urbanization, economic shifts, and nonrenewable energy usage, globalization and the use of sustainable power sources enhance environmental quality over the long-run.

The article "Anthropological responses to environmental challenges in SAARC nations: A comparative analysis" was retracted in 2025. Reasons: concerns about the peer review; concerns about the authorship.

## 5. Conclusions

The study has examined the impact of GDP, ENP, HC, ENS, and REC on LE using a board stationarity data from 1995 to 2022 of SAARC countries. The study has applied the DSK check technique, DH causality test, CSD test, SHL test, board stationarity test, and cointegration test. The results demonstrate that environmentalists and health experts have made LE a principal area because of the ever-increasing waste of non-renewable energy sources. Results show that SAARC countries’ GDP, ENP, and REC are on the right track for future life expectancy growth. Increases in both pollution and reliance on certain financial activities reduce people’s life expectancy. Because the ENS is so bad for HC’s overall government aid and support, the LE eventually fades. The changes in the GDP, the use of green electricity, and public funding are directly related to future improvements inside SAARC countries. A unidirectional relationship between GDP growth, REC, ENS, and LE was found via the causality evaluation test. The results show that higher human resource levels will undoubtedly affect the future, and the human resource improvement is also favorably impacted by a cleaner environment. If SAARC nations are serious about improving public health and environmental sustainability, they must immediately begin to understand the interplay between human capital, environmental degradation, and the future. The study recommends the government officials, scientists, and general health professionals to use the these finds in their advantage in their efforts to reduce pollution and boost environmentally friendly for long-run economic growth. The environment pollution has negative effects on human health, including an increased risk of respiratory infections, cardiovascular problems, and other ailments that harm future generations. To propel future advancements, the SAARC nations’ state-run administrations should put financial growth at the top of their list. More money for research means more opportunities to build cutting-edge hospitals, make life-saving medical equipment more widely available, and create better treatments. The research hopes that by tackling problems like resource distribution, emerging infectious illnesses, regional differences, intervention efficacy, and coordinated evaluation, we can fill in the gaps in our knowledge and be better prepared in the long run. This will help safeguard public health and lessen the effects of pollution on the environment, and it will pave the way for studies to come that will push for policies backed by data.

The article "Anthropological responses to environmental challenges in SAARC nations: A comparative analysis" was retracted in 2025. Reasons: concerns about the peer review; concerns about the authorship.

### 5.1 Future research suggestions

The future is increased by REC speculation, which in turn increases medical care offices and administrations through ventures, businesses, foundations, and development. SAARC countries should prioritize REC agreements and development rules. The study suggests that SAARC countries legalize natural norms; punishing environmental offenders would deter others. To transition away from petroleum derivatives and toward sustainable electricity, the government and its partners are pushing for cleaner energy sources, raising awareness about asset depletion challenges, and launching capital initiatives to improve people’s livelihoods.
